The article "Ultrasonic Intelligent Diagnosis of Papillary Thyroid Carcinoma Based on Machine Learning" was retracted in 2023. Reasons: signs of a paper mill; compromised peer review; unreliable results or conclusions.

# Ultrasonic Intelligent Diagnosis of Papillary Thyroid Carcinoma Based on Machine Learning

**DOI:** 10.1155/2022/6428796

**Published:** 2022-01-10

**Authors:** Heng Zhou, Bin Liu, Yang Liu, Qunan Huang, Wei Yan

**Affiliations:** ^1^Ultrasound Department, Hubei Provincial Hospital of TCM, Wuhan 430061, China; ^2^Network and Computing Center, Huazhong University of Science and Technology, Wuhan 430000, China; ^3^Department of Ultrasound Diagnosis, Central Theater General Hospital of the Chinese People's Liberation Army, Wuhan 430000, China

## Abstract

Thyroid diseases are divided into papillary carcinoma and nodular diseases, which are very harmful to the human body. Ultrasound is a common diagnostic method for thyroid diseases. In the process of diagnosis, doctors need to observe the characteristics of ultrasound images, combined with professional knowledge and clinical experience, to give the disease situation of patients. However, different doctors have different clinical experience and professional backgrounds, and the diagnosis results lack objectivity and consistency, so an intelligent diagnosis technology for thyroid diseases based on the ultrasound image is needed in clinic, which can give objective and reliable diagnosis opinions on thyroid diseases by extracting the texture, shape, and other information of the image and assist doctors in clinical diagnosis. This paper mainly studies the intelligent ultrasonic diagnosis of papillary thyroid cancer based on machine learning, compares the ultrasonic characteristics of PTMC diagnosed by using the new ultrasound technology (CEUS and UE), and summarizes the differential diagnosis effect and clinical application value of the two technology methods for PTMC. In this paper, machine learning, diffuse thyroid image features, and RBM learning methods are used to study the ultrasonic intelligent diagnosis of papillary thyroid cancer based on machine learning. At the same time, the new contrast-enhanced ultrasound (CEUS) technology and ultrasound elastography (UE) technology are used to obtain the experimental phenomena in the experiment of ultrasonic intelligent diagnosis of papillary thyroid cancer. The results showed that 90% of the cases were diagnosed by contrast-enhanced ultrasound and confirmed by postoperative pathology. CEUS and UE have reliable practical value in the diagnosis of PTMC, and the combined application of CEUS and UE can improve the sensitivity and accuracy of PTMC diagnosis.

## 1. Introduction

The adenoid gland is the most important endocrine gland in the human body, which plays a very important role in human metabolism. Thyroid cancer is one of the most common malignant tumors of the endocrine system. Thyroid nodules in 5% ∼ 15% thyroid cancer are malignant. The incidence rate of thyroid cancer is increasing year by year. The incidence rate in women is generally higher than that in men. Papillary thyroid carcinoma is the most common clinical feature of thyroid cancer. It has the characteristics of high differentiation, low malignancy, good prognosis, and long survival. However, local metastasis and distant metastasis can also occur. Studies have shown that the rate of lymph node metastasis in papillary thyroid carcinoma is 84.7%, of which two-thirds have 70% lymph node metastases to thyroid cancer, and the incidence rate of thyroid cancer ranges from 70% to 85%. Local invasion or distant metastasis of thyroid cancer may increase the chance of postoperative recurrence. Therefore, metastasis of thyroid cancer is one of the important factors affecting the prognosis of patients.

The article "Ultrasonic Intelligent Diagnosis of Papillary Thyroid Carcinoma Based on Machine Learning" was retracted in 2023. Reasons: signs of a paper mill; compromised peer review; unreliable results or conclusions.

Early detection of thyroid cancer metastasis can help clinicians to estimate the surgical conditions. Ultrasound is the most important imaging method for the diagnosis of thyroid cancer metastasis, which is not only convenient but also accurate and reliable. With the continuous improvement of instrument performance, high-frequency ultrasound can not only sensitively display the internal structure of lesions but also provide blood flow information or judge the quality of lesions. In 2009, the American Thyroid Association emphasized the significance of ultrasound in thyroid nodules in the diagnosis and treatment manual of thyroid nodules and differentiated thyroid cancer and evaluated the ultrasonic thyroid examination as Grade A. Ultrasound examination is of great significance for early detection of thyroid cancer metastasis, early treatment, and improving the survival rate and quality of life of patients and has an important impact on the prognosis of patients.

The thyroid gland secretes thyroid hormones and reduces them. It is an important endocrine organ in the human body. It can regulate the metabolism of material and energy and affect the growth and development of the human body. The gold standard for clinical diagnosis of thyroid diseases is the examination of biological tissues, which confirms that the research of thyroid has entered the era of “big data.” Current datasets usually involve thousands of different variables, including clinical, neuroimaging, genomics, proteomics, transfer genomics, and other “omics” indicators. Iniesta R believes that the analysis of these datasets is challenging, especially when the number of measurements exceeds the number of individuals and may become more complex due to the lack of highly relevant data on subjects and variables. The statistical learning model is a natural extension of classical statistical methods, but it provides a more effective method for analyzing very large datasets. In addition, the prediction ability of this model is expected to play a role in the development of the decision support system. In other words, methods of clinical setting and guidance, such as diagnostic classification or personalized treatment, can be introduced. This paper discusses the advantages of statistical learning in thyroid research from the perspective of research and clinical practice, but there is a lack of specific data [1]. Jean N believes that there are still some reliable data on economic livelihoods in developing regions, and the problems in these regions can be improved by studying relevant technologies. This shows the correct, cheap, and scalable method of estimating consumption expenditure and assets and properties from high-resolution satellite images. By studying how to train and fold the neural network to recognize the features of the image, these features can show up to 75% of the changes in the first-class economic results. At the same time, it also shows that the powerful machine learning technology can be applied to the limited training data settings and establish a wide range of potential applications in multiscientific fields, but there is a lack of necessary experimental data [2]. Lenoir J believes that a centralized literature review of machine learning (ML) and data mining (DM) methods for network analysis supports intrusion detection. A brief tutorial description of each ML/DM method is provided. According to the number of references or the relevance of emerging methods, we can identify, read, and summarize. Because data are very important in ML/DM methods, some famous network datasets used in ML/DM are introduced. At the same time, the complexity of the ML/DM algorithm, the challenges of using the ML/DM algorithm in network security, and some suggestions on when to use the given method were put forward, but there is a lack of numerical analysis content [3]. Obermeyer Z believes that deep reinforcement learning has been successful in medicine. However, the thyroid will be a challenging task to deal with because of the blurring of characters in visual appearance, such as height or depth. In addition, this kind of action in intelligent medicine usually involves knowledge, which also makes the network design very difficult. An open intelligent medical environment similar to a gym is created, and an A3C + network for learning RL agents is proposed. The model includes a circular information network, which uses the characteristics of intelligent medical information with circular layer to study different diseases. In the experiment, LF2 in different environments is considered, which successfully proves the application of the proposed model in deep learning, but part of the discussion is not accurate enough [4].

The article "Ultrasonic Intelligent Diagnosis of Papillary Thyroid Carcinoma Based on Machine Learning" was retracted in 2023. Reasons: signs of a paper mill; compromised peer review; unreliable results or conclusions.

The innovation of this paper is that machine learning, diffuse image features of the thyroid, and RBM learning methods are used to study the ultrasonic intelligent diagnosis of papillary thyroid cancer based on machine learning. However, the shape, texture, edge, and other information of nodules need to be considered in clinical diagnosis of nodular diseases. Therefore, segmentation and classification research is not independent of each other. We can further explore the influence of artificial features on neural network features.

## 2. Machine Learning Method

### 2.1. Machine Learning

Machine learning is a multidisciplinary discipline, which involves probability theory, statistics, and many other disciplines. Machine learning algorithm is an algorithm that automatically analyzes and obtains rules from data and uses these rules to predict unknown data [5]. At present, it is generally believed that Warren McCulloch and Walter Pitts completed the first work of artificial intelligence in 1943 and proposed the M-P neuron model based on three resources, such as basic physiological knowledge and functional analysis of brain neurons. At the same time, they put forward the formal analysis of logic for Russell, Whitehead, and Turing's computer theory. In 1950, Alan Turing published the book on artificial intelligence, and the concepts of machine learning, genetic algorithm, and reinforcement learning are defined and explained in R&D [6, 7]. In the same year, two Harvard students built the first neural network computer named SNARC, which uses 3000 vacuum tubes and an automatic indicating device to simulate a network composed of 40 neurons [8]. Rosenblatt, an American neuroscientist, proposed the simplest advanced perception of the artificial neural network. Since then, machine learning has made many achievements in the direction of the neural network. In the development of other algorithms, Ross Quinlan, an Australian computer scientist, proposed the famous ID3 algorithm of decision tree. In 1995, Vapnik, a statistician proposed support vector machine, and Freund and Schapire proposed the AdaBoost algorithm [9]. In 2006, Hinton et al. solved the training problem of the deep neural network in the training process, and then, the machine learning developed rapidly and made many achievements. Machine learning is shown in Figure 1.

### 2.2. Thyroid Diffuse Image Features

#### 2.2.1. Statistical Characteristics

Image statistical feature is the overall expression of the characteristics of the image gray distribution, and it is a common feature of the image. In this paper, four features such as gray mean, gray variance, gray third-order moment, and statistical entropy are extracted to express the uniformity of the image gray distribution [10]. For size X, the definition of gray mean value, second-order moment, third-order moment, and statistical entropy of Y image are, respectively, as follows:

(1) $$\begin{array}{c} u=\frac{1}{X\times Y}\sum_{a=1}^{X}\sum_{b=1}^{Y}Q\left(a,b\right),\\ \sigma =\sqrt{\sum_{a=1}^{X}\sum_{b=1}^{Y}{\left[Q\left(a,b\right)-u\right]}^{2}},\\ En=\sum_{i=0}^{255}k_{i}\log\;k_{i}. \end{array}$$

The article "Ultrasonic Intelligent Diagnosis of Papillary Thyroid Carcinoma Based on Machine Learning" was retracted in 2023. Reasons: signs of a paper mill; compromised peer review; unreliable results or conclusions.

#### 2.2.2. Feature Extraction Based on Gray-Level Co-Occurrence Matrix and Gray-Level Run-Length Matrix

In the process of constructing the GLRLM, this paper proposes the longest highlight run feature combined with the GLRL feature, that is, the length of the highest highlight run continuously distributed in the image, as the texture feature of papillary carcinoma [11, 12]. The longest highlight run can represent the stretch and echo-intensity of ultrasonic image texture from the linear structure of image texture:

(2) $$\begin{array}{c} m\text{Long Run}=\max\left(k,h\right). \end{array}$$

where h is the H-th column of the moment GLRL and k is the element binarization and other preprocessing methods in the GLRLM, when the image is decomposed by 2D-DWT. 2D-DWT can be realized for the low-frequency HH sub-image again according to the actual situation [13]. As the texture scale of the ultrasonic image changes greatly, a single-scale wavelet decomposition may miss a lot of image details:

(3) $$\begin{array}{c} HH\left(a,b\right)=i. \end{array}$$

#### 2.2.3. Feature Extraction of Multi Subgraph Co-Occurrence Matrix Based on Multilevel Wavelet

For the *PH* and *HP* subgraphs obtained after a 2D-DWT, the two components retain the coupling information of the high- and low-frequency components in the horizontal and vertical directions, so they can be fused into new subgraphs:

(4) $$\begin{array}{c} \text{PHP}=\sqrt{PH^{2}+HP^{2}}. \end{array}$$

PHP preserves the local and texture information in the original image, which is called the overall detail subimage, considering that the element data range of the first-level wmcm constructed from different images is not necessarily the same, and directly extracting features from the first-level wmcm may have an impact on the subsequent work:

(5) $$\begin{array}{c} h\left(i,j\right)=\frac{h\left(i,j\right)}{\sum_{i=1}^{X}\sum_{j=1}^{Y}h\left(i,j\right)},\\ h\left(i\right)=\sum_{j=1}^{X}h\left(i,j\right). \end{array}$$

After binary, the number of bright areas for the normal and Graves' disease is large and scattered, and they will not be concentrated in a certain area of the image, while the distribution of bright areas for Hashimoto's disease is concentrated on the stripe-like texture of Hashimoto's disease. This method can not only recognize the stripe-like texture of Hashimoto's disease, but also accurately marks all the coverage areas of stripe-like texture, and it is conducive to further analysis [14]. Based on the processed ultrasonic image, the strip feature is defined as follows:

(6) $$\begin{array}{c} h=\frac{\log\left(a+1\right)}{\log\;F_{a}}, \end{array}$$

where *a* is the number of bars and Sn is the area of the highlighted area in the binary graph. The number of highlight areas in different images is different, but the number of highlight areas is generally small due to the existence of the Hashimoto feature. Generally, the highlight area of the image without the stripe feature is larger than that of the image with the stripe feature [4, 15].

The article "Ultrasonic Intelligent Diagnosis of Papillary Thyroid Carcinoma Based on Machine Learning" was retracted in 2023. Reasons: signs of a paper mill; compromised peer review; unreliable results or conclusions.

### 2.3. Ultrasonic Diagnosis

Ultrasound is the most important imaging method in the diagnosis of thyroid cancer metastasis, which is not only convenient but also accurate and reliable. With the continuous improvement and improvement of instrument performance, high-frequency ultrasound can not only sensitively display the internal structure of lesions but also provide blood flow information, so as to judge the benign and malignant lesions [16]. The 2009 guidelines for the diagnosis and treatment of thyroid nodules and differentiated thyroid cancer issued by the American Thyroid Association clearly emphasized the importance of ultrasound examination of thyroid nodules and assessed the importance of ultrasound examination of thyroid as Grade A [17]. Ultrasound plays an important role in the early detection and treatment of thyroid cancer metastasis, improving the survival rate and quality of life of patients and has an important impact on the prognosis of patients, as shown in Figure 2.

With the continuous improvement and improvement of the performance of the ultrasonic diagnostic instrument, the application of high-frequency ultrasound in small organ examination has become an important content of ultrasonic diagnosis, especially for the examination of thyroid diseases. With the advantages of high resolution, high sensitivity, simple operation, and rapid diagnosis, ultrasound has become the preferred method for the examination of thyroid diseases [18, 19]. Especially with the popularization of high-frequency probe, color Doppler, and Doppler spectrum technology, the sensitivity and resolution of ultrasound have been significantly improved. It can not only observe small lesions of 1-2 mm size but also clearly shows the abnormal echo, abnormal blood flow signal, and abnormal blood flow spectrum inside the lesions. It provides a very favorable condition for the early diagnosis of thyroid tumor and peripheral neck lesions.

The article "Ultrasonic Intelligent Diagnosis of Papillary Thyroid Carcinoma Based on Machine Learning" was retracted in 2023. Reasons: signs of a paper mill; compromised peer review; unreliable results or conclusions.

### 2.4. RBM Learning Method

RBM is a model based on the energy function. The energy model first defines the energy function of the whole model and achieves the learning purpose through the energy function. It is assumed that the variables in the visible layer and hidden layer obey the Bernoulli distribution, and the energy function is defined as *l* loss function, which is the most commonly used mean square error function. In some cases, the optimization function needs regularization and density constraints on the values of some parameters to make the learned features more general and avoid the overlapping problem. The common method to increase the density constraint is to introduce the KL entropy. In the self-coding network, by increasing the constraint conditions, the average value of the hidden layer output is limited to 0, so as to reduce the feature. Finally, the optimization function with constraints is as follows:

(7) $$\begin{array}{c} H\left(a,r:e\right)=-\sum_{i=1}^{I}\sum_{j=1}^{J}f_{ij}a_{i}r_{j}, \end{array}$$

where *e* is the RBM parameter and *r* is the connection weight between the visible layer and the hidden layer. In this case, the joint distribution of the visible layer variable *m* and the hidden layer variable *b* is obtained:

(8) $$\begin{array}{c} f\left(m,\frac{h}{e}\right)=\frac{\exp\left(-H\left(a,r:e\right)\right.}{Z}. \end{array}$$

The conditional probability is as follows:

(9) $$\begin{array}{c} f\left(g=\frac{1}{r};e\right)=\sigma \left(\sum_{i=1}^{l}u_{ij}h_{i}+b\right). \end{array}$$

Benign thyroid nodules have clear texture and uniform echo, while malignant thyroid nodules have rough texture and large echo difference. Six features, such as aspect ratio, compactness, rectangular fitting factor, circular area of nodule boundary, and standard deviation of gray scale inside the nodule are used to describe benign thyroid nodules. Therefore, the aspect ratio of benign nodules is generally small. However, when malignant nodules grow, they will invade into adjacent normal tissues, resulting in irregular shape of nodules, so the aspect ratio is generally larger. The definition of the aspect ratio is as follows:

(10) $$\begin{array}{c} F=\frac{H}{L}. \end{array}$$

where *H* is the longest longitudinal diameter and *L* is the longest transverse diameter. Compactness is the expression of the edge features of an object based on the relationship between the area and perimeter of the object:

(11) $$\begin{array}{c} F=\frac{4\pi S}{H^{2}}. \end{array}$$

In which, *S* is the area covered by the nodule area, which can be calculated by the number of pixels included in the nodule area. *H* is the circumference of the nodule. It can be calculated by the number of points included in the nodule edge. The rectangular fitting factor can be expressed by the ratio of the coverage area of the nodule and the minimum outer rectangular coverage area of the nodule:

(12) $$\begin{array}{c} F={\frac{S}{S}}_{\text{rec}}. \end{array}$$

The article "Ultrasonic Intelligent Diagnosis of Papillary Thyroid Carcinoma Based on Machine Learning" was retracted in 2023. Reasons: signs of a paper mill; compromised peer review; unreliable results or conclusions.

## 3. Ultrasound Intelligence-Related Experiments of Papillary Thyroid Carcinoma

### 3.1. Staging Method

Methods: a total of 70 patients with papillary thyroid carcinoma (PTC) were enrolled in the Department of Endocrinology of the First Affiliated Hospital of Medical University. The diameter of the tumor was less than or equal to 10 mm, and the number of lymph nodes was 107. All the patients were confirmed by biopsy. At the same time, pathology and complete medical records (including thyroid ultrasound images and pathological reports) can be collected, so we can analyze and summarize the patient's identity, tumor risk, and new ultrasound technology images horizontally. The data of postoperative disease examination are all analyzed by using SPSS18.0 software; when *p* < 0.05, the difference was statistically significant. According to the imaging characteristics of new ultrasound techniques (CEUS and UE), the characteristics of important parameters related to benign and malignant thyroid nodules were analyzed and compared. The diagnostic effect and related indicators of PTMC were calculated by using statistical principles, and the diagnostic value of main parameters of PTMC was compared.

### 3.2. Objects

In the Department of Endocrinology and Mammary Gland of the First Affiliated Hospital of Medical University and in the electronic medical record system, 70 patients with tumor diameter ≤10 mm and 107 lymph nodes were selected, including 10 male patients and 60 female patients. The medical history ranged from days to years, with an average of 7 months; The average age is 30 years, and the ratio of male to female patients is about 1 : 6, as shown in Table 1.

We collected and analyzed the image information obtained by using the new ultrasound technology and conducted a cross-comparison study on the basic information of patients, tumor characteristics, and the imaging performance of the new ultrasound technology (CEUS and UE) as well as the results of disease examination. The important parameters were sorted out and entered into the Microsoft Excel database. Based on the hardness of the tissue, it can be divided into five grades, as shown in Table 2.

The article "Ultrasonic Intelligent Diagnosis of Papillary Thyroid Carcinoma Based on Machine Learning" was retracted in 2023. Reasons: signs of a paper mill; compromised peer review; unreliable results or conclusions.

### 3.3. Characteristic Manifestations of Contrast-Enhanced Ultrasound

CEUS will start to study all pathologically confirmed thyroid lesions in the following four aspects. The criteria for judging PTMC are uneven low enhancement, early regression, and nonedge enhancement or irregular enhancement, with edge as the criteria for determining PTMC, as shown in Figure 3:

### 3.4. Ultrasonic Examination

As a common clinical auxiliary examination, ultrasound is widely used in the diagnosis of superficial organs such as the thyroid. It is economical, sensitive, safe, and radiation-free. It provides not only the morphology of the tissue but also hemodynamic information. With the development of ultrasound microbubble engineering and biotechnology, some specific ultrasound microbubble contrast agents have been constructed and their value in tumor diagnosis has been gradually explored. Contrast agents are not only imaging agents but also carriers of various molecular markers and drugs. They can be used in proteomics to find the occurrence and development of thyroid cancer-related proteins. At the same time, when differential expression analysis of thyroid tumor protein is combined with an ultrasound targeted lipid microbubble contrast agent, we can realize ultrasound molecular-level imaging and observe the specific binding of the targeted contrast agent to the thyroid cancer tissue at molecular and cellular levels. The targeted ultrasound technology can achieve early diagnosis of papillary thyroid cancer, and this technology can be extended to clinical diagnosis and treatment, which can also be combined with drug-loaded ultrasound microbubble production technology and can provide relevant basis for clinical further development of targeted therapeutic drugs.

## 4. Intelligent Ultrasonic Diagnosis of Papillary Thyroid Carcinoma

### 4.1. Characteristics of Ultrasound

X test was used to compare the different characteristics of CEUS in thyroid micro benign and malignant tumors. Statistical analysis showed that the CEUS enhancement mode, intensity, early retirement, and edge enhancement were significantly different between micro benign and malignant tumors (*p* < 0.05) (67% (65/75), 76.00% (57/75), 85.33% (64/75), and 76). However, most of the benign thyroid microlesions showed homogeneous moderate enhancement (62.50%, 20/32), a few showed high enhancement (15.63%, 5/32), and generally disappeared at the same time or late stage (87.50%, 28/32). Most of them had edge structures, that is, regular edge enhancement signs (75.00%, 24/32), as shown in Table 3:

The following three groups of cells were observed by using targeted microbubbles labeled with monoclonal antibodies and nontargeted lipid microbubbles without labeled monoclonal antibodies under an optical microscope: ① papillary thyroid cancer cells, ② thyroid benign adenoma cells, and ③ normal thyroid cells and the combination of targeted and nontargeted contrast agents in the optical microscope. The third group of normal thyroid cells was the control group, and the optical microscope can see the normal thyroid cells in the control group, and the targeted and nontargeted microbubbles are not bound. The benign adenoma cell group combined with the targeted microbubbles in a small amount but not with the nontargeted microbubbles. The cancer cell group was closely bound with the targeted microbubbles and did not bind with the nontargeted microbubbles. Under a light microscope, the targeted microbubbles of the cancer cell group can be seen closely connected with the peripheral and outer edge of the cell wall of thyroid cancer cells, which indicates that the targeted microbubbles of the cancer cell group are closely associated with thyroid cancer cells as shown in Figure 4.

The article "Ultrasonic Intelligent Diagnosis of Papillary Thyroid Carcinoma Based on Machine Learning" was retracted in 2023. Reasons: signs of a paper mill; compromised peer review; unreliable results or conclusions.

Papillary carcinoma of the thyroid gland may be characterized by widespread fibrous hyperplasia. The stripe feature and the longest highlight run of GLRL have good expression ability for the stripe feature, so they can be used to distinguish different papillary carcinoma images in the feature selection process.

### 4.2. Ultrasonic Elastography Results and Pathological Diagnosis

Among 107 nodules, 75 were malignant and 32 were benign. Among them, 70 cases were with an UE score ≥3, and 5 cases were with an UE score ≤2; In addition, there were 32 benign small thyroid lesions, 21 with an UE score ≤2, and 3 were with an UE score ≥3, as shown in Table 4.

Table 4 shows that the thyroid nodules have various features such as shape and texture. The traditional target segmentation method is only effective for some of the nodes with obvious features, and it is difficult to adapt to a large number of different types of nodules. If artificial design is carried out for a large number of nodules, it will not only increase the complexity of the method but also reduce the robustness of the algorithm and affect the segmentation effect of the target. In addition, a large number of different features are needed to be designed for the diagnosis of benign and malignant nodules. The priority relationship between the strengths and weaknesses of different features is difficult to quantify. Therefore, it is difficult to match with a large number of clinical data, and it is difficult to use the traditional machine learning method to diagnose thyroid nodule diseases.

The article "Ultrasonic Intelligent Diagnosis of Papillary Thyroid Carcinoma Based on Machine Learning" was retracted in 2023. Reasons: signs of a paper mill; compromised peer review; unreliable results or conclusions.

### 4.3. Comparison of Diagnostic Effectiveness of the New Ultrasonic Technology

If three or more possible malignant features appear in ultrasound images, the possibility of nodules is more malignant. Therefore, the shape and texture characteristics of the nodules should be quantitatively characterized for thyroid nodule diseases. The differentiation between benign and malignant thyroid nodules is shown in Table 5:

The region of interest selection principle of thyroid nodular disease image is different from that of papillary thyroid cancer image. Firstly, due to the different sizes of nodules in different patients, the focus depth of ultrasound images is not consistent. If a uniform fixed size ROI is used to extract nodules, it is easy to lose the edge and overall shape information of large nodules. If the ROI size is too large, it is easy to mix too much irrelevant information into the image of small nodules, and it is easy to ignore the details of small nodules, Therefore, the size of ROI needs to be determined according to the size of the nodule and cannot be limited by a fixed size. When selecting the ROI, we should try to make the ROI cover all the areas of the nodules and should keep some areas outside the edge of the nodules, so as to compare the gray changes of the boundary areas of thyroid nodules and the differences between the internal and external areas of the nodules, as shown in Figure 5:

In 90 cases of malignant tumors, 60 cases were correctly diagnosed by CEUS and 30 cases by UE, while in 25 cases of benign tumors, 10 cases were correctly diagnosed by CEUS and 15 cases were correctly diagnosed by UE. In addition, the advantage chi-square comparison results showed that UE had higher sensitivity in the differential diagnosis of thyroid micro benign and malignant nodules, and the difference was significant. Also, through the comparison of the diagnostic specificity between the two, the results show that UE shows greater advantages, and the difference is significant, as shown in Figure 6:

The sensitivity and specificity of CEUS were 85.34% and 67.54%, respectively, while those of UE were 90.21% and 78.45%, respectively. The statistical superiority chi-square analysis showed that UE had higher diagnostic efficiency in the differential diagnosis of PTMC. If combined, the sensitivity and specificity for the diagnosis of thyroid micro benign and malignant nodules can reach 78.43% and 78.67%, respectively.

Referring to the typical reference in the development of machine learning, it marks the data as a class and automatically classifies it into a class. The Bayesian e-mail recognition algorithm is a classification algorithm. In the algorithm design, the corresponding threshold is designed to judge the attributes of an e-mail. If the value obtained from the algorithm is less than this number, it is an ordinary e-mail. If it is higher than this number, it is spam. To ensure the accuracy of the judgment, we must let the system learn the correct threshold experience value through more sample mails and massive intelligent data.

The article "Ultrasonic Intelligent Diagnosis of Papillary Thyroid Carcinoma Based on Machine Learning" was retracted in 2023. Reasons: signs of a paper mill; compromised peer review; unreliable results or conclusions.

## 5. Conclusion

In this paper, machine learning, diffuse thyroid image features, and RBM learning methods are used to study the ultrasonic intelligent diagnosis of papillary thyroid cancer based on machine learning. Through the experiment of ultrasonic intelligent diagnosis of papillary thyroid cancer, the new ultrasonic technology (CEUS and UE) is used to get the experimental phenomenon. The onset of papillary thyroid cancer is more hidden in the early stage, and there were no obvious symptoms and signs. Some studies found that the early regional lymph node metastasis rate was 50% ∼ 80%, and the early distant organ metastasis rate was about 10%. Papillary thyroid cancer needs to be diagnosed in time and treated (mainly by surgical lobectomy, supplemented by thyroid stimulating hormone inhibitor). Most patients can be cured, and the survival rate is high. However, in practice, early and accurate diagnosis of thyroid cancer is difficult. At present, the judgment of benign and malignant thyroid nodules is based on the comprehensive results of the patient's history, color Doppler ultrasound, CT, fine-needle aspiration smear, and intraoperative frozen tissue section. Among them, B-ultrasound-guided fine-needle aspiration and intraoperative fast frozen tissue section are the important basis for the diagnosis of thyroid cancer, which is of great significance for the selection of treatment plan, operation mode, and prognosis of patients. With the development of ultrasound diagnosis technology, it provides a new idea for clinical diagnosis and treatment, which is a new treatment technology for papillary thyroid cancer. Although with the development of new technology, there are still many problems to be solved in the application of this technology in papillary thyroid cancer and circulatory system diseases. There are no serious problems in the sustainability of scientific and technological development, and ultrasonic intelligent diagnosis technology is of great significance to the clinical diagnosis and treatment of human diseases, as it provides a new and more accurate method for disease diagnosis and treatment.

## Figures and Tables

**Figure 1:** Machine learning.

**Figure 2:** Contrast-enhanced ultrasound of the thyroid (http://alturl.com/nmmj2).

The article "Ultrasonic Intelligent Diagnosis of Papillary Thyroid Carcinoma Based on Machine Learning" was retracted in 2023. Reasons: signs of a paper mill; compromised peer review; unreliable results or conclusions.

**Figure 3:** Performance of characteristic phenomena.

**Figure 4:** Papillary thyroid carcinoma (http://alturl.com/ntod7).

**Figure 5:** Multivariate analysis of potential risk factors for T staging of esophageal cancer.

**Figure 6:** Comparison of new ultrasound techniques in the diagnosis of thyroid micro benign and malignant nodules.

**Table 1:** Research objects.

Information	Quantity
Male patients	10
Female patients	60
Medical History	7
Age	30
Male to female ratio	1 : 6

**Table 2:** Evaluation criteria.

Color	Fraction	Scale
Red, blue, and green	0	0
Green	1	100%
Green	2	>90%
Blue and green	3	60% ∼ 90%
Blue	4	>90%

**Table 3:** Contrast-enhanced ultrasonography of thyroid nodules.

CEUS performance	Malignant	Benign
Inhomogeneous enhancement	70	8
Low enhancement	60	10
Early fade	50	5
Regular annular enhancement	20	30

**Table 4:** Comparison of ultrasound elastography of different thyroid micro benign and malignant nodules.

Pathological type	UE	CEUS
Malignant	75	15
Benign	32	24
X	75.43	26.54
P	0.02	0.03

**Table 5:** The main reference factors of ultrasound in the diagnosis of benign and malignant thyroid nodules.

	Benign	Malignant
Composition	Pure cystic	Pure solid
Shape	Regular	Irregular
Boundary	Clear	Not clear

## Data Availability

The simulation experiment data used to support the findings of this study are available from the corresponding author upon request.
